# An E2F5-TFDP1-BRG1 Complex Mediates Transcriptional Activation of MYCN in Hepatocytes

**DOI:** 10.3389/fcell.2021.742319

**Published:** 2021-10-22

**Authors:** Zhiwen Fan, Ming Kong, Xiulian Miao, Yan Guo, Haozhen Ren, Jinglin Wang, Shuai Wang, Ning Tang, Longcheng Shang, Zhengyi Zhu, Hanyi Liu, Wei Zhu, Xiaolei Shi

**Affiliations:** ^1^Department of Hepatobiliary Surgery, Affiliated Nanjing Drum Tower Hospital of Nanjing University Medical School, Nanjing, China; ^2^Hepatobiliary Institute, Nanjing University, Nanjing, China; ^3^Key Laboratory of Targeted Intervention of Cardiovascular Disease, Collaborative Innovation Center for Cardiovascular Translational Medicine, and Center for Experimental Medicine, Department of Pathophysiology, Nanjing Medical University, Nanjing, China; ^4^College of Life Sciences and Institute of Biomedical Research, Liaocheng University, Liaocheng, China; ^5^Department of Anesthesiology, The Affiliated Drum Tower Hospital of Nanjing University Medical School, Nanjing, China

**Keywords:** transcriptional regulation, hepatocyte, liver regeneration, epigenetics, chromatin remodeling protein, proliferation

## Abstract

Liver regeneration is characterized by cell cycle reentrance of hepatocytes. N-Myc, encoded by MYCN, is a member of the Myc family of transcription factors. Elevation of MYCN expression has been noted in the course of liver regeneration whereas the underlying mechanism remains unclear. Here we describe that up-regulation of MYCN expression, as measured by quantitative PCR, Western blotting, and immunohistochemical staining, paralleled liver regeneration in animal and cell models. MYCN expression was up-regulated as a result of transcriptional activation. Ingenuity pathway analysis (IPA) revealed several up-stream transcriptional regulators for MYCN and RNA interference validated E2F5 and TFDP1 as essential for hepatocyte growth factor (HGF)-induced MYCN *trans*-activation. Further examination showed that deficiency of BRG1, a chromatin remodeling protein, attenuated MYCN induction during liver regeneration. BRG1 interacted with and was recruited by E2F5/TFDP1 to the MYCN promoter. Mechanistically, BRG1 might play a role regulating histone H3 acetylation and H3K4 trimethylation and facilitating/stabilizing the binding of RNA polymerase II surrounding the MYCN promoter. Over-expression of ectopic MYCN in BRG1-null hepatocytes overcame deficiency of proliferation. Importantly, a positive correlation between MYCN expression and BRG1/E2F5/TFDP1 expression was observed in human liver specimens. In conclusion, our data identify a novel epigenetic pathway where an E2F5-TFDP1-BRG1 complex regulates MYCN transcription to promote liver regeneration.

## Introduction

Exposed to various injuries stimuli including surgical resection, pathogens, corrosive chemicals, toxins, and ischemia/anoxia, hepatocytes undergo necrosis or apoptosis leading to the loss of liver parenchyma and consequently liver function. A regenerative response may ensue in which quiescent hepatocytes re-enter the cell cycle and resume proliferation to compensate for the loss of liver mass and function (Fausto et al., 2006). Defective liver regeneration is often associated with poor prognosis in patients with end-stage liver disease (ESLD) and liver failure. On the contrary, vigorous liver regeneration contributes to the normalization of liver function after injury and predicts better outcome in ESLD patients (Forbes and Newsome, 2016). During the process of liver regeneration, a complex hierarchy of regulatory factors, including growth factors, signaling molecules, and transcription factors, cooperate to enable quiescent hepatocytes to progress through different checkpoints of cell cycle, to re-acquire the ability to undergo mitosis and to replicate (Kurinna and Barton, 2010, 2011). For instance, the E2F family of transcription factors, typically functioning as an E2F-TFDP dimer, is compulsive for hepatocytes to leap through the G1/S transition (Trimarchi and Lees, 2002). E2F deletion impairs the spatiotemporal control of liver regeneration in mice whereas deficiency in E2F activity has been found to be responsible for aging-induced weakening of liver regenerative capacity (Trimarchi and Lees, 2002; Delgado et al., 2011).

MYC represents a family of proto-oncoproteins that all contain a basic helix-loop-helix (bHLH) DNA binding domain. Three members, C-MYC (encoded by MYCC), N-MYC (encoded by MYCN), and L-MYC (encoded by MYCL), have been identified for the MYC family (Meyer and Penn, 2008). As transcription factors, MYC proteins bind to the consensus E-box (CACGTG) sequence located on their target promoters and regulate the expression of genes involved in cell growth, differentiation, and death (Pellanda et al., 2021). There has been a large body of research work documenting the role of MYC proteins in the regulation of liver regeneration. The Fausto laboratory was among the first to report that C-MYC up-regulation in hepatocytes is an early event following partial hepatectomy (Goyette et al., 1984). Consistently, C-MYC transgenic mice exhibit significant advantage in terms of liver regenerative response over the wild type littermates after the surgical resection (Factor et al., 1997). In addition, high C-MYC expression is associated with better prognosis in patients after the surgical removal of hepatocellular carcinoma likely owing to heightened regenerative potential (Ji et al., 2018). Mechanistic studies have found that the Wnt-β-catenin signaling cascade is primarily responsible for C-MYC up-regulation at the transcriptional level in proliferating hepatocytes during liver regeneration (Yang et al., 2008). Huber et al. (1989) examined the levels of poly-A^+^ mature message RNAs in hepatocellular carcinomas (HCC) of different grades in rats: whereas c-MYC expression was clearly correlated with the proliferative potential of HCC cells, no L-MYC or N-MYC expression was detected. Recently, several studies have found that L-MYC gene polymorphism may be associated with altered susceptibility to HCC development and progression but it remains unclear whether L-MYC could directly regulate hepatocyte proliferation and, if so, what the mechanism might be (Taylor et al., 1993; Hsieh et al., 1996; Park et al., 2002). Comparatively more is known regarding the role of N-MYC in the regulation of hepatocyte proliferation than L-MYC. Elevation of N-MYC expression in the regenerating livers has also been reported although the underlying transcriptional mechanism is not entirely clear (Corral et al., 1988).

Brahma-related gene 1 (BRG1) is a chromatin remodeling protein playing versatile roles in hepatic pathophysiological processes including non-alcoholic steatosis (Fan et al., 2020; Kong et al., 2021c), fulminant hepatitis (Hong et al., 2021), liver fibrosis (Dong et al., 2020), and septicemic injury (Dong et al., 2021). BRG1 down-regulation is associated with hepatocyte differentiation during liver development (Inayoshi et al., 2005). In contrast, BRG1 deletion in the adult liver blocks hepatocyte proliferation after partial hepatectomy (Li et al., 2019; Wang et al., 2019). Of note, hepatic c-MYC expression was down-regulated in the BRG1 conditional knockout (CKO) mice compared to the WT mice (Li et al., 2019). Because Corral et al. (1988) have demonstrated that MYCN expression could be induced in the proliferating livers following hepatectomy, we hypothesized that BRG1 might contribute to MYCN up-regulation. In the present report we identify MYCN as a novel transcriptional target for BRG1 in hepatocytes. Mechanistically, BRG1 interacts with E2F5 and TFDP1 and directly binds to the MYCN promoter to activate MYCN transcription in response to pro-regenerative stimuli. In addition, re-introduction of MYCN into BRG1-null hepatocytes corrects the deficiency of proliferation. More importantly, a positive correlation between MYCN expression and BRG1/E2F5/TFDP1 expression is observed in human liver specimens. Therefore, targeting the E2F5/TFDP1-BRG1-MYCN axis may prove effective in the treatment of liver failure.

## Materials and Methods

### Animals

All animal protocols were reviewed and approved the intramural Ethics Committee on Humane Treatment of Laboratory Animals of Nanjing Medical University. The mice were maintained in an SPF environment with 12 h light/dark cycles and libitum access to food and water. Hepatocyte conditional Brg1 knockout (Brg1^LKO^) mice have been described previously (Kong et al., 2021a). Liver injury was induced by intraperitoneal injection of acetaminophen (APAP) or ischemia-reperfusion as previously described (Li et al., 2019). Briefly, APAP was dissolved in 1XPBS and the mice received a single injection at a dose of 300 mg/kg. Alternatively, the mice were anesthetized with ketamine/xylazine and laparotomy was performed down the midline to expose the liver. An atraumatic clip was placed across the portal vein, hepatic artery, and bile duct to block blood flow. After 90min of ischemia, the clip was removed and the abdomen was closed with suture. The mice were euthanized by pentobarbital sodium (100–120 mg/kg) at indicated time points following APAP injection or reperfusion.

### Cells, Transient Transfection, and Reporter Assay

Primary murine hepatocytes were isolated as previously described (Kong et al., 2021b). Mouse recombinant HGF was purchased from R&D. The cells were treated with HGF (20 ng/ml) for 12–48 h as indicated. BRG1 expression construct has been previously described (Li et al., 2020). MYCN promoter-luciferase construct was generated by amplifying genomic DNA spanning the proximal promoter and the first exon of MYCN gene (−225/ + 18) and ligating into a pGL3-basic vector (Promega). Mutagenesis was performed a QuikChange kit (Thermo Fisher Scientific, Waltham, MA, United States). All DNA constructs were verified by direct sequencing. Small interfering RNAs were purchased from GenePharma: siFoxp2, CGAAUUUUAUAAAAACGCA; siFoxp1, GCAGGCGGTACTCAGACAAAT; siTwist2, AC AGUAAGAAGUCGAGCGAAGAUGG; siE2f5, GUUCGUGU CGCUGCUGCAGTT; siTfdp1, GGAGACTTGAAAGAATAAA. Cells were harvested 24–48 h after the transfection. Transient transfections were performed with Lipofectamine 2000. Luciferase activities were assayed using a luciferase reporter assay system (Promega) as previously described (Zhang et al., 2021).

### Protein Extraction and Western Blot

Whole cell lysates were obtained by re-suspending cell pellets in RIPA buffer (50 mM Tris pH7.4, 150 mM NaCl, 1% Triton X-100) with freshly added protease inhibitor (Roche) as previously described (Yang et al., 2021). Western blot analyses were performed with anti-MYCN (Proteintech, 10159-2), anti-BRG1 (Abcam, Ab110641), anti-E2F5 (Thermo Fisher, PA5-81166), anti-TFDP1 (Thermo Fisher, PA5-86135), anti-FOXP1 (Abcam, ab227649), anti-FOXP2 (Abcam, ab16046), anti-TWIST2 (Abcam, ab66031), and anti-β-actin (Sigma, A1978). For densitometrical quantification, densities of target proteins were normalized to those of β-actin as previously described (Liu et al., 2021b). Data are expressed as relative protein levels compared to the control group which is arbitrarily set as 1.

### RNA Isolation and Real-Time PCR

RNA was extracted with the RNeasy RNA isolation kit (Qiagen) as previously described (Liu et al., 2021a). Reverse transcriptase reactions were performed using a SuperScript First-strand Synthesis System (Invitrogen) as previously described (Chen et al., 2021). Real-time PCR reactions were performed on an ABI Prism 7500 system with the following primers: *Mycn*, 5′-ACCATGCCGGGGATGATCT-3′ and 5′-AGCATCTCCGTAGCCCAATTC-3′; *Ccna2*, 5′-TGGATGGCAGTTTTGAATCACC-3′ and 5′-CCCTAAGGTA CGTGTGAATGTC-3′; *Ccne1*, 5′-CTCCGACCTTTCAGTCC GC-3′ and 5′-CACAGTCTTGTCAATCTTGGCA-3′; *Ccnb1*, 5′-CAATTATCGGAAGTGTCGGATCA-3′ and 5′-CTGGTGAACGACTGAACTCCC-3′; *Pcna*, 5′-TTT GAGGCACGCCTGATCC-3′ and 5′-GGAGACGTGAGA CGAGTCCAT-3′. Ct values of target genes were normalized to the Ct values of housekeekping control gene (18s, 5′-CGCGGTTCTATTTTGTTGGT-3′ and 5′-TCGTCTTCGAAACTCCGACT-3′ for both human and mouse genes) using the ΔΔCt method and expressed as relative mRNA expression levels compared to the control group which is arbitrarily set as 1 as previously described (Zhang et al., 2020).

### Chromatin Immunoprecipitation

Chromatin Immunoprecipitation (ChIP) assays were performed essentially as described before (Wu et al., 2020). In brief, chromatin in control and treated cells were cross-linked with 1% formaldehyde. Cells were incubated in lysis buffer (150 mM NaCl, 25 mM Tris pH 7.5, 1% Triton X-100, 0.1% SDS, 0.5% deoxycholate) supplemented with protease inhibitor tablet and phenylmethylsulfonyl fluoride (PMSF). DNA was fragmented into ∼200 bp pieces using a Branson 250 sonicator. Aliquots of lysates containing 200 μg of protein were used for each immunoprecipitation reaction with anti-BRG1 (Abcam, ab110641), anti-E2F5 (Thermo Fisher, PA5-81166), anti-TFDP1 (Thermo Fisher, PA5-86135), anti-acetyl H3 (Millipore, 06–599), anti-trimethyl H3K4 (Millipore, 17–614), anti-RNA polymerase II (Abcam, ab264350), anti-p300 (Abcam, ab275378), anti-KMT2A (Bethyl laboratories, A300-087A), or pre-immune IgG. Precipitated DNA was amplified with the following primers: 5′-AGGCTTTTCCCCGCCCTC-3′ and 5′-AGAGAGAGAGAGTCGGAAAAAAG-3′.

### Histology

Histological analyses were performed essentially as described before (Li et al., 2021). Paraffin sections were stained with were blocked with 10% normal goat serum for 1 h at room temperature and then incubated with anti-MYCN (Proteinch, 1:200) or anti-PCNA (Abcam, 1:200) antibodies. Staining was visualized by incubation with anti-rabbit secondary antibody and developed with a streptavidin-horseradish peroxidase kit (Pierce) for 20 min. Pictures were taken using an Olympus IX-70 microscope. Quantifications were performed with Image J.

### Ingenuity Pathway Analysis

Ingenuity pathway analysis (IPA) was performed using “MYCN” as keyword with the proprietary software developed by Qiagen (Hilden, Germany) per vendor instructions.

### Human Acute Liver Failure Specimens

Liver biopsies were collected from patients with ALF referring to Nanjing Drum Tower Hospital. Written informed consent was obtained from subjects or families of liver donors. All procedures that involved human samples were approved by the Ethics Committee of the Nanjing Drum Tower Hospital and adhered to the principles outlined in the Declaration of Helsinki. Paraffin sections were stained with indicated antibodies.

### 5-Ethynyl-2′-Deoxyuridine Incorporation Assay

5-ethynyl-2′-deoxyuridine (EdU) incorporation assay was performed in triplicate wells with a commercially available kit (Thermo Fisher) as previously described (Wu et al., 2021). Briefly, the EdU solution was diluted with the culture media and incubated with the cells for 2 h at 37°C. After several washes with 1XPBS, the cells were then fixed with 4% formaldehyde and stained with Alexa Fluor^TM^ 488. The nucleus was counter-stained with DAPI. The images were visualized by fluorescence microscopy and analyzed with Image-Pro Plus (Media Cybernetics). For each group, at least six different fields were randomly chosen and the positively stained cells were counted and divided by the number of total cells. The data are expressed as relative EdU staining compared to the control group arbitrarily set as 1.

### Statistical Analysis

One-way ANOVA with *post hoc* Scheff’e analyses were performed by SPSS software (IBM SPSS v18.0, Chicago, IL, United States). Unless otherwise specified, values of *p* < 0.05 were considered statistically significant.

## Results

### MYCN Up-Regulation Parallels Hepatocyte Proliferation *in vivo* and *in vitro*

Of the three MYC family members, the regulatory role of c-MYC in liver regeneration has been extensively studied whereas little is known regarding the expression patterns of L-MYC in hepatocytes or its regulation. On the other hand, Corral et al. (1988) have reported that N-MYC expression is up-regulated during liver regeneration in a rat model of partial hepatectomy but the underlying mechanism is unclear. Therefore, we focused our study on the regulatory mechanism that might contribute to N-MYC up-regulation in proliferating hepatocytes. We examined the fluctuation of MYCN expression in the course of liver regeneration in two different animal models. In the first model, the mice were injected with a single dose of acetaminophen (APAP) to induce acute liver injury; liver regeneration typically peaks between 12 h and 48 h after the injection (Bhushan and Apte, 2019). Quantitative PCR showed that MYCN mRNA levels started to increase 12 h following APAP injection, peaked at 24 h, and declined at 48 h (Figure 1A); the pattern of MYCN expression tracked closely with hepatocyte proliferation as indicated by proliferating cell nuclear antigen (PCNA) expression. Protein levels of MYCN, as measured by Western blotting (Figure 1B) and immunohistochemical staining (Figure 1C), were similarly up-regulated and mirrored the kinetics of hepatocyte proliferation. In an alternative model, the mice were subjected to 45 min of hepatic ischemia followed by reperfusion; liver regeneration occurs as early as a few hours after the injury and can sustain for a couple of days (Schlossberg et al., 1996; Martins and Markmann, 2013). As shown in Figures 1D–F, there was again a simultaneous up-regulation of MYCN and the proliferative marker PCNA during the hepatic regenerative response as assessed by qPCR, Western blotting, and immunohistochemical staining. Finally, when primary murine hepatocytes were exposed to the pro-proliferative growth factor HGF, it was discovered that MYCN expression was strongly up-regulated by HGF treatment (Figures 1G,H).

**FIGURE 1:** MYCN up-regulation parallels hepatocyte proliferation *in vivo* and *in vitro*. **(A–C)** C57B6/L mice were injected with APAP (300 mg/kg) and sacrificed at indicated time points. MYCN expression was examined by qPCR, Western blotting, and immunohistochemical staining. **(D–F)** C57B6/L mice were subjected to ischemia-reperfusion and sacrificed at indicated time points. MYCN expression was examined by qPCR, Western blotting, and immunohistochemical staining. **(G,H)** Primary murine hepatocytes were treated with HGF and harvested at indicated time points. MYCN expression was examined by qPCR and Western. Data are expressed as mean ± standard deviation (SD). *p<0.05 (one-way ANOVA with *post hoc* Scheffe test).

### Hepatocyte Growth Factor Induced MYCN Transcription Requires an Intact E2F Site

To verify whether the observed induction of MYCN expression during liver regeneration was due to altered transcription rate, a *MYCN* promoter-luciferase construct (−225/ + 18) was transfected into HepG2 cells followed by HGF treatment. The *MYCN* promoter activity was significantly augmented by HGF treatment as early as 6 h and remained high by 24 h (Figure 2A). In order to uncover the upstream transcriptional regulators that might mediate MYCN induction by HGF, we performed ingenuity pathway analysis (IPA), which revealed the top five putative regulators of MYCN transcription to be FOXP2, E2F5, TFDP1, TWIST2, and FOXP1 (Figure 2B). To further narrow the specific regulator(s) of MYCN transcription, siRNAs targeting each individual transcription factor were designed, transfected into murine primary hepatocytes, and validated by Western blotting (Figure 2C). Knockdown of E2F5 or TFDP1 was sufficient to attenuate HGF-induced MYCN expression at mRNA (Figure 2D) and protein (Figure 2E) levels where knockdown of the other three factors did not impact MYCN expression. E2F5 and TFDP1 belong to the E2F family of transcription factors that recognize the consensus TTTSSCGC motif (La Thangue, 1994). To further demonstrate the essentiality of E2F5/TFDP1 in MYCN transcription, two putative E2F sites (TTGGCGCG) located on the proximal MYCN promoter, one between −181 and −174 relative to the transcription start site and the other between −162 and −155, were mutated and the mutant promoter displayed significantly weakened response to HGF treatment (Figure 2F).

**FIGURE 2:** HGF induced MYCN transcription requires an intact E2F site. **(A)** A MYCN promoter-luciferase construct was transfected into HepG2 cells followed by treatment with HGF. The cells were harvested at indicated time points and luciferase activities were normalized by GFP fluorescence and protein concentration. **(B)** IPA analysis of upstream regulators of MYCN. **(C)** Primary murine hepatocytes were transfected with indicated siRNAs. Knockdown efficiencies were verified by Western. **(D,E)** Primary murine hepatocytes were transfected with indicated siRNAs followed by treatment with HGF for 24 h. MYCN expression was examined by qPCR and Western. **(F)** WT or mutant MYCN promoter-luciferase construct was transfected into HepG2 cells followed by treatment with HGF for 24 h. Luciferase activities were normalized by GFP fluorescence and protein concentration. Data are expressed as mean ± standard deviation (SD). *p<0.05 (one-way ANOVA with *post hoc* Scheffe test).

### MYCN Down-Regulation as a Result of Hepatocyte Conditional BRG1 Deletion

BRG1 is a chromatin remodeling protein playing essential roles in liver regeneration (Li et al., 2019; Wang et al., 2019). We asked whether BRG1 might be involved in the regulation of MYCN transcription. To this end, WT and BRG1 hepatocyte conditional knockout (CKO) mice were injected with APAP and sacrificed 24 h later. As shown in Figure 3A, compared to the APAP-injected WT livers, MYCN mRNA expression in the APAP-injected CKO livers was down-regulated by 72%. Western blotting (Figure 3B) and immunohistochemical staining (Figure 3C) showed a decrease in MYCN protein expression in the CKO livers compared to the WT livers. Similarly, in the ischemia-reperfusion model, BRG1 deficiency repressed MYCN expression in the livers as measured by qPCR (Figure 3D), Western blotting (Figure 3E), and immunohistochemistry (Figure 3F). When primary hepatocytes were isolated from WT and BRG1 CKO mice and treated with or without HGF, MYCN induction was much less prominent in the CKO cells than in the WT cells (Figures 3G,H). Finally, the MYCN promoter-luciferase construct was transfected into WT and CKO cells followed by HGF treatment; augmentation of the *MYCN* promoter activity by HGF treatment in the CKO cells was not as strong as in the WT cells (Figure 3I), pointing to the mandatory role of BRG1 in MYCN transcription.

**FIGURE 3:** MYCN down-regulation as a result of hepatocyte conditional BRG1 deletion. **(A–C)** WT and BRG1 CKO mice were injected with APAP (300 mg/kg) and sacrificed 24 h after the injection. MYCN expression was examined by qPCR, Western blotting, and immunohistochemical staining. **(D–F)** WT and BRG1 CKO mice were subjected to ischemia-reperfusion and sacrificed 24 h after the injection. MYCN expression was examined by qPCR, Western blotting, and immunohistochemical staining. **(G,H)** Primary murine hepatocytes were isolated from WT and BRG1 CKO mice and treated with or without HGF for 24 h. MYCN expression was examined by qPCR and Western. **(I)** A MYCN promoter-luciferase construct was transfected into primary murine hepatocytes isolated from WT and BRG1 CKO mice followed by treatment with HGF. The cells were harvested at indicated time points and luciferase activities were normalized by GFP fluorescence and protein concentration. Data are expressed as mean ± standard deviation (SD). *p < 0.05 (one-way ANOVA with *post hoc* Scheffe test).

### BRG1 Interacts With E2F5-TFDP1 to Activate MYCN Transcription

We next examined the potential interplay between BRG1 and E2F5/TFDP1 in regulating MYCN transcription. Co-immunoprecipitation assay showed that BRG1 could form a complex with both E2F5 and TFDP1 in primary hepatocytes (Figure 4A). Chromatin immunoprecipitation (ChIP) assay showed that in response to HGF treatment, the occupancies of E2F5, TFDP1, and BRG1 on the MYCN promoter region were similarly increased and followed the kinetics of MYCN expression (Figure 4B). Depletion of endogenous E2F5 or TFDP1 largely abrogated the binding of BRG1 to the MYCN promoter suggesting that BRG1 might rely on its interaction with E2F5/TFDP1 to bind to the MYCN promoter (Figure 4C). The binding of either E2F5 or TFDP1, on the other hand, was not reciprocally influenced by each other (Figures 4D,E). Since E2F5 or TFDP1 appears to be non-redundantly necessary for MYCN *trans*-activation and for BRG1 recruitment to the MYCN promoter, it is likely that E2F5 and TFDP1 may form a dimmer and cooperatively recruit BRG1, which serves as a rate-limiting factor for MYCN *trans*-activation; loss of either component of this complex would disrupt BRG1 binding and consequently dampen MYCN *trans*-activation.

**FIGURE 4:** BRG1 interacts with E2F5-TFDP1 to activate MYCN transcription. **(A)** Immunoprecipitation was performed with anti-BRG1 or IgG using primary murine hepatocyte lysates. **(B)** Primary murine hepatocytes were treated with HGF and harvested at indicated time points. ChIP assays were performed with anti-BRG1, anti-E2F5, anti-TFDP1, or IgG. Upper panel, a scheme of the MYCN promoter highlighting the positions of the two proximal E2F sites and the ChIP primers. TSS, transcription start site. **(C–E)** Primary murine hepatocytes were transfected with indicated siRNAs followed by treatment with HGF. ChIP assay was performed with anti-BRG1, anti-E2F5, and anti-TFDP1. **(F–L)** Primary hepatocytes were isolated from WT and BRG1 CKO mice followed by treatment with HGF. ChIP assays were performed with anti-E2F5, anti-TFDP1, anti-acetyl H3, anti-trimethyl H3K4, anti-RNA polymerase II, anti-p300, and anti-KMT2A. Data are expressed as mean ± standard deviation (SD). *p < 0.05 (one-way ANOVA with *post hoc* Scheffe test).

On the contrary, recruitment of either E2F5 or TFDP1 to the MYCN promoter did not appear to be reliant on BRG1 because E2F5/TFDP1 binding on the MYCN promoter was comparable in the WT cells and the CKO cells (Figures 4F,G). When the WT cells were exposed to HGF, histone H3 acetylation (Figure 4H) and H3K4 trimethylation (Figure 4I) started to abound the MYCN promoter consistent with transcriptional activation. The changes in acetyl H3 and trimethyl H3K4 surrounding the MYCN promoter were much subtler in the CKO cells. In addition, the recruitment of RNA polymerase II was severely compromised in the absence of BRG1 likely explaining the reduced transcription rate (Figure 4J). Because previous studies have suggested that BRG1 can interact with histone acetyltransferase p300 (Xu et al., 2015) and histone H3K4 methyltransferase KMT2A (also known as mixed lineage leukemia 1, MLL1) (Shao et al., 2020), we hypothesized that BRG1 might recruit p300 and/or KMT2A to the MYCN promoter to alter histone modifications. ChIP assays performed with anti-p300 (Figure 4K) and anti-KMT2A (Figure 4L) antibodies showed that occupancies of both enzymes on the MYCN promoter were up-regulated by HGF treatment, which were weakened by BRG1 deficiency.

### MYCN Over-Expression Overcomes BRG1 Deficiency and Normalizes Hepatocyte Proliferation

In order to further demonstrate the functional relevance of BRG1-dependent MYCN transcription in hepatocyte proliferation, a rescue experiment was performed. Adenovirus carrying either MYCN (Ad-MYCN) or GFP (Ad-GFP) was used to transduce primary hepatocytes isolated from WT or BRG1 CKO mice. As shown in Figures 5A,B, expression levels of several cell cycle regulators involved in hepatocyte proliferation, including cyclin A2 (Ccna2), cyclin B1 (Ccnb1), and cyclin E1 (Ccne1) were down-regulated in the CKO cells compared to the WT cells. Over-expression of ectopic MYCN, however, partially restored the expression of the cell cycle regulators. In addition, EdU incorporation assay showed that HGF-induced hepatocyte proliferation was impaired in the CKO cells, which could be corrected by MYCN over-expression (Figure 5C).

**FIGURE 5:** MYCN over-expression overcomes BRG1 deficiency and normalizes hepatocyte proliferation. **(A–C)** Primary hepatocytes were isolated from WT and BRG1 CKO mice and transduced with adenovirus carrying MYCN expression vector followed by treatment with HGF. Gene expression levels were examined by qPCR and Western. Cell proliferation was measured by EdU staining. **(D)** Human ALF specimens were stained with indicated antibodies. Linear regression was performed with Graphpad Prism. Data are expressed as mean ± standard deviation (SD). *p < 0.05 (one-way ANOVA with *post hoc* Scheffe test).

Finally, we compared the correlation between MYCN and its upstream regulators in human liver specimens. As shown in Figure 5D, MYCN expression was stronger in the liver with higher levels of BRG1/E2F5/TFDP1. Linear regression analysis identified significant correlation between MYCN expression and BRG1/E2F5/TFDP1 expression (Figure 5D).

## Discussion

Liver regeneration is programmed by multiple pro-proliferative transcription factors, the levels of which undergo dynamic changes in the process (Taub, 1996; Costa et al., 2003; Kurinna and Barton, 2011; Colak et al., 2020). N-Myc (MYCN), a member of the Myc family of proto-oncoproteins, is transcriptionally up-regulated in the proliferating livers (Corral et al., 1988). Here we detail a novel mechanism whereby the chromatin remodeling protein BRG1, *via* interacting with E2F5 and TFDP1, regulates MYCN transcription in hepatocytes in response to pro-proliferative stimuli. In addition, MYCN over-expression partially corrects the deficiency of proliferation in BRG1-null hepatocytes. The direct *in vivo* evidence that supports a causal relationship between MYCN and liver regeneration is lacking at this point. Mice homologous for *Mycn* deletion die prematurely during embryogenesis with defects in several major organs including the heart, the brain, the gut, and the lungs (Charron et al., 1992; Stanton et al., 1992; Sawai et al., 1993) thus precluding the analysis of liver regeneration in these animals. However, studies exploiting spatiotemporally conditional MYCN knockout (CKO) mice clearly support a pro-proliferative role for MYCN *in vivo*. For instance, Harmelink et al. (2013) have reported that MYCN deletion in the myocardium, by crossing the *Mycn*^f/f^ mice to the *cTnt*-Cre mice, results in a failure in ventricular wall morphogenesis; the CKO mice display significantly reduced proliferation rate of cardiomyocyte with concomitant down-regulation in *Ccnd1* and *Ccnd2*. Likewise, Dominguez-Frutos et al. (2011) have shown that MYCN deletion in the inner ear (*via* crossing the *Mycn*^f/f^ mice to the *Pax2*-Cre mice) causes hearing defects owing to diminished proliferation of the otic vesicle. These observations do not automatically foretell the role of MYCN in liver regeneration because several independent investigations have concluded that hepatocyte-specific deletion of c-Myc, whose expression is similarly up-regulated during liver regeneration as MYCN, minimally influences liver regeneration after partial hepatectomy in mice (Baena et al., 2005; Li et al., 2006; Sanders et al., 2012). It is possible that different Myc proteins may play redundant roles in liver regeneration wherein the loss of one Myc factor could be fully compensated by others. New animal studies, by crossing the *Mycn*^f/f^ mice to the *Alb*-Cre mice for instance, would hopefully solve this lingering issue.

Through IPA and validation studies, we identify E2F5 and TFDP1 as the key transcription factors that recruit BRG1 to activate MYCN transcription. Unlike the “activating” E2Fs that include E2F1, E2F2, and E2F3, E2F5 is typically considered a transcriptional repressor although it possesses a similar *trans-*activating (TAD) domain (Trimarchi and Lees, 2002). However, there is evidence to support E2F5 as a transcriptional activator (Fry et al., 1997; Teissier et al., 2010; Xie et al., 2020). It remains unclear whether our finding that E2F5 activates MYCN expression represents a norm or an exception for its role as a transcription regulator. Of note, BRG1 knockdown dampens the presence of active histone modifications on the MYCN promoter and hampers the recruitment of RNA polymerase II suggesting that E2F5 may rely on its interaction with BRG1 to function as an activator of transcription. Equally uncertain is the implication of this finding in liver regeneration *in vivo*. Mice with germline E2F5 deletion (*E2f5*^–/–^) are born with Mendelian ratio essentially ruling out a role for E2F5 in embryogenesis. However, the *E2f5*^–/–^ mice die before reaching adulthood due to excessive cerebrospinal fluid production and consequently non-obstructive hydrocephalus (Lindeman et al., 1998). Similarly, TFDP1 deficient mice (*Tfdp1*^–/–^) die during the early extra-embryonic stage in development (Kohn et al., 2003). Clearly new model animals harboring hepatocyte-conditional deletion of E2F5 or TFDP1 are needed in order to clarify their respective roles in MYCN transcription and liver regeneration.

Our data seem to convey a message that boosting the activity of the E2F5-TFDP1-BRG1-MYCN axis could promote liver regeneration and thus mitigate liver failure. However, this potential benefit should be weighed against the risk of malignant transformation. Aberrant activation of MYCN, for instance, has been frequently linked to the development of neuroblastoma, retinoblastoma, leukemia, and, more recently, hepatocellular carcinoma (Rickman et al., 2018; Qin et al., 2018). Thus, an inevitable yet intriguing question to ask is whether or not this E2F5-TFDP1-BRG1-MYCN axis could differentiate signals that instigate physiological hepatocyte proliferation (i.e., liver regeneration) and those that stimulate pathological hepatocyte proliferation (i.e., liver cancer). Further investigations are warranted so that affective and safe therapeutic strategies can be devised to enhance liver regeneration and restore liver function in patients with liver failure.

## Data Availability Statement

The original contributions presented in the study are included in the article/supplementary material, further inquiries can be directed to the corresponding author/s.

## Ethics Statement

The animal study was reviewed and approved by Nanjing Medical University Ethics Committee on Humane Treatment of Experimental Animals.

## Author Contributions

XS and WZ conceived the project and secured the funding and provided the supervision. ZF and MK designed the experiments. ZF, MK, XM, YG, HR, JW, LS, and ZZ performed the experiments and collected data. All authors contributed to the manuscript writing/editing.

## Conflict of Interest

The authors declare that the research was conducted in the absence of any commercial or financial relationships that could be construed as a potential conflict of interest.

## Publisher’s Note

All claims expressed in this article are solely those of the authors and do not necessarily represent those of their affiliated organizations, or those of the publisher, the editors and the reviewers. Any product that may be evaluated in this article, or claim that may be made by its manufacturer, is not guaranteed or endorsed by the publisher.
